The article "Association of Sarcopenia and Low Nutritional Status with Unplanned Hospital Readmission after Radical Gastrectomy in Patients with Gastric Cancer: A Case-Control Study" was published in 2022. Journal: J Healthc Eng.

# Association of Sarcopenia and Low Nutritional Status with Unplanned Hospital Readmission after Radical Gastrectomy in Patients with Gastric Cancer: A Case-Control Study

**DOI:** 10.1155/2022/7246848

**Published:** 2022-04-15

**Authors:** Yiqi Cai, Shan Chen, Xiaodong Chen, Wenjing Chen, Pengfei Wang, Guanbao Zhu, Jinji Jin

**Affiliations:** ^1^Department of Gastrointestinal Surgery, The First Affiliated Hospital of Wenzhou Medical University, Wenzhou, China; ^2^First Clinical College of Wenzhou Medical University, Wenzhou, China

## Abstract

**Objective:**

Sarcopenia is one of the influencing factors of poor prognosis in patients with gastric cancer but the association with readmission are unknown. We aimed to explore factors associated with readmission after gastrectomy and to determine whether preoperative sarcopenia is a common outcome in readmitted patients.

**Methods:**

In this case-control study, patients who underwent gastric resection in the First Affiliated Hospital of Wenzhou Medical University between April 2016 and September 2017 were included. The reasons of readmission patients were described. The readmission patients and non-readmission patients were matched by propensity score matching (PSM). The univariate analysis was applied for the baseline characteristics, operative details, postoperative prognosis and discharge disposition, and multiple logistic regression analysis for the independent risk factors of readmission.

**Results:**

The unplanned readmission rate within 30 days of radical gastrectomy for gastric cancer was 6.5% (43/657). The average time interval from discharge to readmission was 13 days. Delayed gastric evacuation was the main cause of readmission (18.6%, 8/43). Body mass index (BMI), nutritional risk screening (NRS) 2002 score, history of abdominal surgery, sarcopenia, and preoperative albumin were included in the multivariate logistic regression analysis. NRS 2002 (OR = 3.43, 95% CI: 1.10–10.72, *P*=0.034) and sarcopenia (OR = 4.25, 95% CI: 1.13–16.02, *P*=0.033) were found to be independently associated with unplanned readmission within 30 days of radical gastrectomy for cancer. Other factors such as age, sex, BMI, American Society of Anesthesiologists grade, surgical method, operation and reconstruction type, TNM stage, surgical duration, previous abdominal surgery, and preoperative albumin and hemoglobin level were not associated with unplanned readmission after radical gastrectomy for cancer.

**Conclusions:**

Sarcopenia and low nutritional status are independently associated with unplanned readmission within 30 days of radical gastrectomy for cancer.

## 1. Introduction

Unplanned readmission refers to readmission of patients in a short duration due to the same or related illness after discharge. Unplanned readmission exacerbates the patient's physical and mental stress, prolongs the hospitalization time, increases the treatment cost, and overburdens medical resources, so has been receiving increasing attention [1, 2]. In 2004, readmission-related medical expenses in the United States reached $17.4 billion [1]. Moreover, unplanned readmission has become an important indicator for evaluating the quality of medical care worldwide [1].

According to GLOBOCAN 2018 [3], based on the incidence, gastric cancer is the fourth most common malignant tumor; while based on the mortality, gastric cancer ranks third. In China, approximately 410,000 new cases of gastric cancer are reported every year [4, 5], accounting for 42% of cases worldwide [3]. Gastrectomy remains the gold-standard treatment for gastric carcinoma [6, 7]. However, the patients who have undergone gastrectomy often develop postoperative complications, and unplanned readmissions have become common in the patients [8, 9]. Previous studies have examined the incidence rate and related factors of readmission after surgeries for colorectal and hepato-pancreato-biliary cancers [10–17]; however, those have not been studied in the case of gastric cancer.

Gastric resection is a complicated surgery associated with high postsurgical morbidity and mortality [18]. A study reported that unplanned readmission is associated with increased mortality of patients who undergo radical gastrectomy [19]. However, the factors associated with readmission after radical gastrectomy have not been studied. Identification of the influencing factors for readmission after radical gastrectomy can help prevent readmission and improve the management of patients with gastric cancer.

tSarcopenia refers to progressive age-related loss of skeletal muscles and their function, resulting in weakness [20]. Sarcopenia can be prevented by regular physical activity, healthy diet including adequate intake of carbohydrates and proteins, and the maintenance of body weight in the normal range [21]. Sarcopenia is not only associated with falls, physical frailty, functional disability/loss of independence, and increased risk of mortality [20], but also correlated with the risk of poor outcomes after major surgeries [22–26]. At present, many current studies have shown that preoperative sarcopenia is associated with the postoperative risks for the complications, mortality, and length of hospital stay after gastrointestinal tumor surgery [27–29]. However, the correlation between sarcopenia and postoperative readmission in patients with gastric cancer has not been reported.

Therefore, the objective of this study was to explore factors associated with readmission after gastrectomy, and to determine whether preoperative sarcopenia is a common outcome in readmitted patients.

## 2. Materials and Methods

### 2.1. Study Design and Samples

This study was a retrospective case-control study that included the patients who underwent elective gastric resection for p-stages I-III primary gastric cancer in the Department of Gastrointestinal Surgery of The First Affiliated Hospital of Wenzhou Medical University between April 2016 and September 2017. The patients were managed according to the Japanese gastric cancer treatment guidelines 2014 [30].

The inclusion criteria were shown as follows: (1) age≥18 years; (2) diagnosis of gastric cancer; and (3) discharge from the hospital after successful elective gastrectomy and reconstruction surgery. The exclusion criteria were displayed as follows: (1) death within 30 days after discharge from the hospital; (2) palliative surgery; (3) patients with residual gastric cancer or concomitant tumor in another organ or system; (4) patients who received neoadjuvant chemotherapy; and (5) patients without sufficient data.

The ethics committee of the First Affiliated Hospital of Wenzhou Medical University approved this study (approval number: 2014 No. 063) and informed consent was obtained from all study participants.

### 2.2. Data Collection

The data were obtained from medical charts and the hospital information system (The data included inpatient number, age, sex, body mass index (BMI), sarcopenia, previous abdominal surgery, preoperative hemoglobin, preoperative albumin, nutritional risk screening (NRS), American Society of Anesthesiology score, surgical approach, type of resection, type of reconstruction, duration of surgery, TNM stage, and major postoperative complications). Based on the Clavien–Dindo grading system, major postoperative complications were defined as grade III or IV [31], including anastomotic leakage, bleeding, failure of conservative drug treatment, adhesive intestinal obstruction, and internal hernia. Unplanned readmission was defined as any emergent hospitalization within 30 days after discharge from the hospital, according to past readmission-related trials [32, 33]. Elective hospital admission for adjuvant therapy was not considered as unplanned readmission in this study. In the case of patients who were hospitalized for multiple physical signs, the most prominent sign was considered as the reason for readmission.

All patients were routinely followed up every 10 days by telephone or outpatient visit for 30 days. Nutritional risk assessment was performed prior to surgery was carried out 24 h after admission according to the NRS 2002 guidelines; the assessment of individuals ≧3 points were considered to be at nutritional risk [33, 34].

### 2.3. Assessment of Sarcopenia

1. Assessment of muscle: Routine preoperative abdominal computed tomography scan was performed in all patients. Lumbar vertebra (L3) imaging was selected for measurement from the Picture Archiving and Communication System (PACS). According to EWGSOP2, muscle area and mean muscle attenuation were utilized to represent muscle quantity and muscle quality, respectively. Muscle was analyzed at computed tomography (CT) workstation (GE ADW 4.5) using specific Hounsfield units (HU) thresholds of -29 to 150, and tissue boundaries were manually outlined as needed. And L3 cross-sectional muscle area was normalized with the square of stature and reported as skeletal muscle index (SMI, cm^2^/m^2^). Cutoff values of SMI were 34.9 cm^2^/m^2^ for females and 40.8 cm^2^/m^2^ for males [35]. The sex-specific cutoff values for mean muscle attenuation in HU of the cross-sectional muscle area were 28.6 HU for females and 38.5 HU for males [35].
2. Muscle strength and physical performance Grip strength and 6 m usual gait speed were tested routinely prior to surgery for the diagnosis of sarcopenia [36, 37]. Myodynamia and physical performance were recorded using an electronic handgrip dynamometer (EH101; Zhongshan Camry Electronic Co., Ltd., Guangdong Province, China). Each subject was allowed to use a dominant hand for all the tests. The 6-m usual gait speed was determined as follows: the patient was allowed to walk over 6 m, and the time from the first footfall to the last one was recorded. The two examinations were completed within 7 days prior to surgery. Additionally, each test was performed three times, and the maximum score was selected [38].
3. Diagnosis of sarcopenia: According to EWGSOP2, sarcopenia was suspected in presence of low muscle strength, and this suspicion was confirmed by documentation of reduced muscle mass or low muscle quality.  Table 1 showed the diagnostic process following the algorithm [35]. To prevent potential ethnic confounders [36, 37], the following criteria were set for the diagnosis of sarcopenia: (1) low SMM (L3 skeletal muscle index <40.8 cm^2^/m^2^ in males and <34.9 cm^2^/m^2^ in females); (2) low myodynamia (handgrip strength <26 kg for males or <18 kg for females); and (3) low muscle performance (6 m usual gait speed <0.8 m/s) [38].

### 2.4. Statistical Analysis

All analyses were performed using SPSS 22.0 (IBM, Armonk, New York, US). Continuous variables were tested for normal distribution by the Kolmogorov–Smirnov test. Moreover, continuous data were presented as means±standard deviations or as medians and interquartile ranges. Normally distributed continuous data were analyzed through the Student's *t*-test. Categorical data were presented as the numbers and percentages and analyzed by the chi-square test. To identify factors associated with readmission within 30 days, the univariate analysis was applied for analyzing baseline characteristics, operative details, postoperative prognosis, and discharge disposition. Multivariate logistic regression analysis was performed with the backward method. Propensity score matching (PSM) was performed for matching readmitted patients with those who were not readmitted. Age and sex were adopted for PSM; matching tolerance was set at 0.05. A *P* value < 0.05 was considered statistically significant.

## 3. Results

### 3.1. Patient Characteristics

Among 710 included patients admitted between April 2016 and December 2017, 697 individuals were eligible for this study. Of the 683 study participants, 7 were excluded because of death within 30 days of discharge, 11 patients because of palliative surgery, 8 patients because of residual gastric cancer or concomitant tumor in another organ or system. In addition, 5 individuals were excluded for receiving neoadjuvant chemotherapy and 9 for insufficient data. Eventually, 657 patients were enrolled in this study (Figure 1) who underwent gastrectomy for cancer, without loss to follow-up. The demographic data and clinical features of the patients were presented in Table 2. Average patient age was 64.5 years, and maximum of the cases (494, and 75.2%) were males. Overall, 43 patients (6.54%) were readmitted within 30 days of discharge. The average time interval from discharge to readmission was 13 days, which was the same as the time interval from readmission to the second discharge. There was no second readmission within 30 days of surgery.

Before PSM, the readmission group had higher NRS (*P*=0.001) and increased rate of major complications (*P* < 0.001) and sarcopenia (*P*=0.001) compared with the patients who were not readmitted.

After PSM, the readmission group had higher NRS (*P*=0.001) and rate of sarcopenia (*P*=0.001), and lower albumin level (*P*=0.010) than the patients who were not readmitted (Table 2).

### 3.2. Reasons for Readmission

Table 3 presents the reasons for readmission. Delayed gastric evacuation was the main reason, accounting for 18.6% of all readmitted patients (8/43). Of the 43 readmitted individuals, 41 received conservative therapy, and two required reoperation, including one each for abdominal internal hemorrhage and gastrointestinal hemorrhage. Besides, two patients diagnosed with anastomotic stricture underwent endoscopic balloon dilation. One of the patients died during readmission because of multiple organ dysfunction syndrome.

### 3.3. Factors Associated with Readmission

The factors associated with readmission were analyzed using the univariate analysis (Table 4). BMI, NRS 2002 score, history of abdominal surgery, sarcopenia, and preoperative albumin were included in the multivariate logistic regression analysis (Table 4). NRS 2002 (OR = 3.43, 95% CI: 1.10–10.72, *P*=0.034) and sarcopenia (OR = 4.25, 95% CI: 1.13–16.02, *P*=0.033) were independently associated with 30-day readmission after radical gastrectomy for cancer.

## 4. Discussion

Unplanned readmission after radical gastrectomy for cancer indicates the threat to patient health because of the high mortality rate in those patients [19, 39]. Sarcopenia is a common condition associated with a high surgical risk [22–26]. Therefore, the identification of factors associated with unplanned readmission after gastric cancer resection is important for the prevention and management of the disease like sarcopenia. For one thing, the frequency of unplanned readmission within 30 days was found to be 6.5%. For another, regression analysis displayed the correlation of sarcopenia and a preoperative NRS 2002 score of ≥3 with readmission within 30 days of radical gastrectomy. These findings showed that sarcopenia and increased NRS score could be considered as indicators of preoperative examination.

Sarcopenia, determined by both muscle quality and quantity, is exacerbated by a poor nutritional status. Age-related sarcopenia is a syndrome associated with progressive and general loss of SMM and myodynamia [36]. Recent reports suggest that sarcopenia is associated with postoperative complications, malnutrition, and unfavorable outcomes in patients with gastric cancer [33, 36]. Besides, sarcopenia is also associated with poor outcomes after major surgeries [22–26]. In this study, sarcopenia was found to be correlated with readmission. Among 657 patients, 19.6% had sarcopenia, and the percentage was consistent with the previous literature [40]. According to this study and our previous studies [33], sarcopenia was highly associated with unplanned readmission. Moreover, the association between sarcopenia and unplanned readmission was also observed in patients who had underwent esophagectomy [25] or abdominoperineal resection [41], as well as in elderly patients in acute care wards [42]. Since sarcopenia can be detected conveniently and objectively, preoperative examination and treatment can be performed to avoid unplanned readmission.

Malnutrition occurs in 36%–43% of patients with gastric cancer, representing a common problem in these individuals [43, 44]. Malnutrition is usually considered a risk for postoperative complications in patients undergoing major abdominal surgery [45, 46]. Currently, many researches have indicated that postoperative complications are the risk factors of unplanned readmission [18, 47, 48]. However, in this study, it is found that postoperative complications were not associated with unplanned readmission. In fact, most of patients with gastric cancer treated at our center who develop postoperative complications were cured during hospitalization before discharge. Therefore, the probability of readmission was greatly reduced in patients with postoperative complications. Also, the above may the reason why there was no significant difference for major postoperative complications in the readmission and non-readmission groups. Our previous study reported that the NRS score of >3 could be considered a risk factor for unplanned readmission of patients after radical gastrectomy [33]. Nevertheless, various subjective factors may affect this score.

The correlation between sarcopenia and readmission after gastrectomy for gastric cancer can be explained by the reflection of SSM on the patient's nutritional status and the association of nutritional risk and postoperative complications as well as readmission [49]. Also, the above explains why sarcopenia is the factor associated with readmission after gastric cancer resection. To a large extent, maintenance of physical function, daily activities, and vitality depends on skeletal muscle strength [49]. Patients with sarcopenia gradually experience weakness and limited mobility, affecting the postoperative recovery process. Therefore, examining the pathogenesis of sarcopenia may help predict the chances in readmission after surgery. Sarcopenia is also associated with postoperative infection and complications [23], which may also explain, at least to some extent, the relationship between sarcopenia and readmission after gastrectomy.

CT is considered as a gold standard for assessing SMM [22]. In clinical practice, patients with gastric cancer routinely receive CT scan for the determination of the size and location of tumors and detection of metastasis. Patients would not incur additional cost or would not be exposed to additional radiation in CT for assessing SSM. The above is applied widely for assessing skeletal muscle quality in patients with gastrointestinal cancer. Therefore, the preassessment of sarcopenia by the surgeon before operation and optimization of the nutritional status of malnourished patients as early as possible are essential.

Gastrointestinal complications such as delayed gastric evacuation, followed by postoperative infectious complications, are the most common causes of readmission, according to previous studies [18, 47]. Majority of patients with sarcopenia face nutritional problems before resection. Specifically, gastrointestinal complications are exacerbated because of lower tolerance to malnutrition. Furthermore, sarcopenia correlates with the high morbidity of infectious complications after operation [45, 46], perhaps contributing to the relationship between sarcopenia and readmission after gastrectomy. In addition, Shi et al. [26] reported that sarcopenia is associated with adverse outcomes after gastrectomy, including longer hospital stay and severe complications. Lieffers et al. [24] reported that sarcopenia is correlated with infection, the need for rehabilitation, and prolonged hospital stay after surgery for colorectal cancer. The management of patients with sarcopenia must focus on the early provision of enteral/parenteral nutrition, nutritional status improvement, and reduction of complications of postoperative intestinal intolerance. All the above can reduce the rate of unplanned readmission.

Combined with the results of our study, we recommended that clinicians not only needed to assess the tumor condition but also needed to evaluate nutritional status and sarcopenia presence of patients. Then, interventions were recommended based on specific diseases and nutritional requirements to improve postoperative outcomes. Combined with the progress of others' studies [28], we recommend treating the application of a high-protein diet or TPN for the treatment of patients with sarcopenia before performing surgical resection. But even so, in the current study, sarcopenia remained an important predictor of clinical outcome.

Whether prolonged postoperative hospitalization contributes to readmission is a highly debatable topic. Kim et al. [47] reported that longer postoperative hospitalization is a critical predictive factor of readmission. Conversely, Ahmad et al. [18] reported that postoperative hospitalization has no significant effect on readmission. In this study, we analyzed the length of first hospital stay after gastrectomy as a categorical (defining 13 days as a cutoff) and continuous variable; and in both the cases, prolonged hospital stay was not associated with readmission within 30 days.

This study has some limitations. First, this was a single-centered study, and the sample size of the readmission group was small. Stronger scientific evidence supported by multicenter prospective studies was needed to confirm these results. Second, we only concluded correlative factors of readmission following gastrectomy within 30 days. Studying the data over a longer term would provide a correlation between the probability of readmission and mortality. Third, as enhanced recovery after surgery (ERAS) was not universally promoted, these results could not be directly applied for all patients with gastric cancer, especially those receiving ERAS. Hence, further investigation was required. Fourth, we did not quantitatively measure the data about food intake, appetite, weight change, and physical activity level.

In conclusion, this study has shown that the rate of readmission within 30 days of radical gastrectomy is 6.5%. A preoperative NRS 2002 score of ≥3 and the occurrence of sarcopenia are associated with the unplanned readmission of patients who have undergone gastrectomy for cancer. Optimization of nutrition, especially in patients with nutritional risk before surgery, can potentially reduce the rate of readmission.

## Figures and Tables

**Figure 1:** Flow chart of the patient screen.

**Table 1:** EWGSOP2 criteria for the diagnosis of sarcopenia.

Probable sarcopenia is identified by criterion 1. Diagnosis is confirmed by additional documentation of criterion 2.
If criteria 1, 2, and 3 are all met, sarcopenia is considered severe
(1) Low muscle strength
(2) Low muscle quantity or quality
(3) Low physical performance

**Table 2:** Characteristics of the readmission and non-readmission groups before and after propensity score matching.

Variable		Before matching			After matching		
		Readmission group (*n* = 43)	Non-readmission group (*n* = 614)	*P*	Readmission group (*n* = 43)	Non-readmission group (*n* = 43)	*P*
Age, years, *n* (%)				0.148			0.110
	<65	25 (58.1)	287 (46.7)		25 (58.1)	32 (74.4)	
	≥65	18 (41.9)	327 (53.3)		18 (41.9)	25 (58.1)	
Sex, male, *n* (%)		32 (74.4)	462 (75.2)	0.904	32 (74.42)	25 (58.1)	0.110
BMI, kg/m^2^, *n* (%)				0.086			0.162
	<18.5	7 (16.3)	48 (7.8)		7 (16.3)	3 (7.0)	
	18.5–23.9	20 (46.5)	378 (61.6)		20 (46.5)	16 (37.2)	
	≥23.9	16 (37.2)	188 (30.6)		16 (37.2)	24 (55.8)	
NRS 2002 score, *n* (%)				0.001			0.001
	<3	15 (34.9)	370 (60.3)		15 (34.9)	33 (76.7)	
	≥3	28 (62.1)	244 (39.7)		28 (62.1)	10 (23.3)	
ASA grade, *n* (%)				0.362			0.059
	I	7 (16.3)	78 (12.7)		7 (16.3)	7 (16.3)	
	II	25 (58.1)	432 (70.4)		25 (58.1)	33 (76.7)	
	III	11 (25.6)	102 (16.6)		11 (25.6)	3 (7.0)	
	IV	0	2 (0.3)		0	0	
Preoperative hemoglobin (g/L)		127 ± 21	119 ± 21	0.435	127 ± 21	131 ± 14	0.251
Preoperative albumin (g/L)		38.5 ± 5.7	37.9 ± 4.6	0.516	38.5 ± 5.7	41.2 ± 3.6	0.010
Surgical approach, *n* (%)				0.702			0.159
	Open surgery	33 (76.7)	455 (74.1)		33 (76.7)	27 (62.8)	
	Laparoscopy	10 (23.3)	159 (25.9)		10 (23.3)	16 (37.2)	
Type of resection, *n* (%)				0.208			0.268
	Subtotal gastrectomy	24 (55.8)	401 (65.3)		24 (55.8)	29 (67.4)	
	Total gastrectomy	19 (44.2)	213 (34.7)		19 (44.2)	14 (32.6)	
Type of reconstruction, *n* (%)				0.190			0.190
	Roux-en-Y	23 (53.5)	253 (41.2)		23 (53.5)	16 (37.2)	
	Billroth I	8 (18.6)	106 (17.3)		8 (18.6)	20 (46.5)	
	Billroth II	12 (27.9)	255 (41.5)		12 (27.9)	7 (16.3)	
TNM stage, *n* (%)				0.735			0.684
	Tis	0	6 (1.0)		0	0	
	I	15 (34.9)	201 (32.7)		15 (34.9)	15 (34.9)	
	II	7 (16.3)	135 (22.0)		7 (16.3)	10 (23.3)	
	III	21 (48.8)	270 (44.0)		21 (48.8)	18 (41.9)	
	IV	0	2 (0.3)		0	0	
Previous abdominal surgery, *n* (%)		9 (20.9)	66 (10.8)	0.075	9 (20.9)	3 (7.0)	0.062
Duration of surgery, *n* (%)				0.068			0.596
	<3.0 hours	8 (18.6)	196 (31.9)		8 (18.6)	10 (23.3)	
	≥3.0 hours	35 (81.4)	418 (68.1)		35 (81.4)	33 (76.7)	
Major postoperative complication, *n* (%)	Grade III or IV	24 (55.8)	168 (27.4)	<0.001	24 (55.8)	28 (65.1)	0.051
Sarcopenia, *n* (%)		25 (58.1)	118 (19.2)	0.001	25 (58.1)	8 (18.6)	0.001

BMI: body mass index; NRS: nutritional risk score; ASA: American Society of Anesthesiologists score.

**Table 3:** Causes of readmission in 43 patients after gastrectomy for gastric cancer.

Causes of readmission	*n* (%)
Delayed gastric emptying	8 (18.60)
Small bowel obstruction	5 (11.62)
Abdominal pain	3 (6.98)
Wound infection	5 (11.62)
Abdominal infection	2 (4.65)
Intra-abdominal hemorrhage	5 (18.10)
Intra-abdominal ﬂuid collection	3 (6.98)
Cholecystitis	2 (4.65)
Gastrointestinal hemorrhage	2 (4.65)
Secondary malignant tumor	2 (4.65)
Deep venous thrombosis	2 (4.65)
Cerebral infarction	1 (2.32)
Pneumonia	1 (2.32)
Appendicitis	1 (2.32)
MODS	1 (2.32)
Total	43

**Table 4:** Univariate and multivariate analyses (backward) of factors potentially associated with readmission in patients with gastric cancer.

Variable	Univariate			Multivariate		
	OR	95% CI	*P*	OR	95% CI	*P*
Age	2.095	0.839–5.227	0.113			
Sex, male, *n* (%)	2.095	0.839–5.227	0.113			
BMI, *n* (%)	0.534	0.278–1.028	0.060	0.540	0.252–1.157	0.113
NRS 2002 score, *n* (%)	6.160	2.393–15.855	0.001	3.429	1.097–10.724	0.034
ASA grade, *n* (%)	1.800	0.831–3.899	0.136			
Surgical approach, *n* (%)	0.522	0.200–1.309	0.162			
Type of resection, *n* (%)	1.640	0.682–3.942	0.269			
Type of reconstruction, *n* (%)	0.775	0.436–1.377	0.384			
TNM stage, *n* (%)	1.092	0.679–1.757	0.716			
Comorbidities, *n* (%)	1.537	0.244–9.695	0.647			
Previous abdominal surgery, *n* (%)	3.529	0.884–14.090	0.074	2.935	0.591–14.584	0.188
Duration of surgery, *n* (%)	1.326	0.467–3.767	0.597			
Major postoperative complication	1.586	0.681–3.737	0.282			
Sarcopenia, *n* (%)	5.031	1.899–13.328	0.014	4.249	1.127–16.015	0.033
Preoperative hemoglobin (g/L)	0.986	0.961–1.010	0.250			
Preoperative albumin (g/L)	0.882	0.797–0.975	0.014	2.935	0.591–14.584	0.652

BMI: body mass index; NRS: nutritional risk score; ASA: American Society of Anesthesiologists score; OR: odds ratio; CI: confidence interval.

## Data Availability

The data used to support the findings of this study are available from the corresponding author upon request.
